The article "Reset and Integration of Music Instructional Resources Using Deep Convolutional Neural Networks" was retracted in 2023. Reasons: signs of a paper mill; suspected computer-generated content; unreliable results or conclusions; concerns about the data.

# Reset and Integration of Music Instructional Resources Using Deep Convolutional Neural Networks

**DOI:** 10.1155/2022/4545125

**Published:** 2022-07-13

**Authors:** Huiling Lei

**Affiliations:** Hunan First Normal University, Changsha 410205, China

## Abstract

In order to overcome the problem that learners and teachers cannot find instructional resources to meet their needs and information overload in the massive resources, this article proposes and designs a music instructional resource management platform based on DCNN. This article expounds the overall goal, design principle, overall structure, and interface design of the system. At the same time, the whole construction process of a music instructional resources integration system based on DCNN is discussed in detail from the aspects of configuration of development environment, localization of platform interface, and realization of main functions of the system. In addition, through the demand analysis tool, the demand of college music instructional resources management is analyzed in detail and deeply, and the demand document is formed. This article makes an in-depth study on the categories of music instructional resources and summarizes the resource classification methods that are in line with the actual instructional activities. The experiments show that the accuracy of the proposed algorithm is improved by about 6% compared with the fuzzy clustering algorithm. At the same time, the stability of this system can reach 96.14%. This system is rich in functions and easy to use and can provide a feasible scheme for the management of instructional resources in various disciplines.

## 1. Introduction

In recent years, the large-scale application of online learning environment has promoted the increasing demand of learners for online instructional resources, resulting in the explosive growth of the number of online instructional resources. Today, with the tide of informatization, the instructional resources in the institution of higher learning have stepped into the era of digitalization and informatization and networking [1]. The continuous development of modern information technology provides more and more information resources for music teaching. How to better develop and utilize these information resources is an important issue that modern music educators have to think about. With the deepening of educational informatization, the information resources in the Internet are increasing exponentially. These resources are not only diverse in content, but also colorful in form [2]. Its impact and penetration in the field of education has made the use of online education resources pay attention, and a new instructional model has emerged. However, at present, the massive online instructional resources have also brought about a serious problem of “information overload.” It is difficult for learners to accurately find out the resources that meet their needs among a large number of instructional resources. At the same time, quality education is a model of modern education and a template for the innovation of talent training mode in higher education. It is of turning significance in the history of music teaching that higher music teaching adheres to the road of quality education. It not only deepens the thought of music teaching, but also makes great progress in exploring the practice of music education. Therefore, it is necessary to reset and integrate music instructional resources and quickly filter irrelevant instructional resources to guide learners to find suitable instructional resources.

All educational resources can be developed and used in order to stimulate students' interest in learning English and improve their aesthetic ability, as long as they can achieve the overall goal of school music curriculum construction. As a result, it is critical to talk about how online educational resources are being developed and integrated. With the advancement of information technology, more textbook resources are being combined into original paper textbooks, and composite textbooks are receiving more attention. The network music education resources cover a wide range of knowledge and content from various disciplines, demonstrating not only the breadth and depth of network resources, but also their ability to disseminate advanced music instructional ideas and methods, as well as music education values and advanced music culture. Application and management of educational resources are at the heart of education informatization. Artificial intelligence [3, 4] is a branch of science that studies how to use various automata to simulate some of human thought processes and intelligent behaviours in order to create intelligent artificial products. The goal of deep learning (DL) [5, 6] as a new machine learning research field is to figure out how to extract multilayer features from data automatically. CNN (convective neural network) [7] is a popular and well-known model in deep learning. The term “neural network” refers to a system in which the input layer's retrieval target provides feedback to the output layer's retrieval results, allowing the output layer to output the corresponding retrieval results. Feedback information is sent to the input layer in this type of network, which is used to store a pattern sequence. The NN style educational resource management system combines the four distinct functions of educational resource storage, educational resource management, educational resource classification, and dynamic upgrading to comprehensively solve the problem of insufficient application in the current basic education informatization process. The music instructional resource platform is built and applied using a DCNN (deep convolution neural network) in this article. The main contributions of this article are as follows:

1. In order to improve the quality of music teaching in the institution of higher learning, this article puts forward some suggestions on effectively resetting and integrating music instructional resources; at the same time, a music instructional resource management platform based on DCNN is proposed and designed. In this article, the algorithm makes use of the advantages of multilayer perceptron in nonlinear data processing and changes the prediction mode of vector multiplication of learner characteristics and instructional resource characteristics into the mode of input multilayer perceptron, thus improving the traditional NN model.
2. The instructional resource integration method realized by DCNN technology in this article is to develop Arduino device identification program by DCNN technology. In the process of learning, learners use Arduino device identification program to obtain instructional resources related to devices and then carry out learning. At the same time, through the demand analysis tool, the demand of music instructional resources management in institution of higher learning is analyzed in detail and deeply, and the demand document is formed. This article makes an in-depth study on the categories of music instructional resources and summarizes the resource classification methods that are in line with the actual instructional activities. The research shows that this method can promote the effective use of music education resources.

## 2. Related Work

In recent years, the integration and recommendation of online instructional resources has become an important research hotspot. Therefore, a large number of scholars in academic circles have conducted extensive research in this direction.

In order to improve the quality of music teaching in the institution of higher learning, Ferguson J R and others put forward suggestions for effectively relocating and integrating music instructional resources, and discussed from three aspects: clarifying educational goals, integrating instructional resources, and innovating college music instructional models [8]. Harrison expounds the concept, types, and characteristics of online music education resources, then presents the results of the online questionnaire survey on both teaching and learning, and mainly analyzes the demand trends of online music education resource service objects [9]. Kuebel analyzes the development and integration of online music education resources from three aspects: the characteristics of online music education resources, the current situation of online music education resources construction, and the development and integration of online music education resource libraries [10]. Bonneville-Roussy and others pointed out that understanding the true meaning of quality education, redeveloping instructional resources for music courses, and optimizing and integrating teaching materials inside and outside the school are the guarantees for the implementation of music quality education in institution of higher learning [11]. Wang et al. proposed an online resource recommendation technology that covers the differences in learning styles, knowledge levels, and learning modes of different learners to overcome the information overload problem that learners have difficulty retrieving instructional resources that meet their needs [12]. Ottone et al. tried to use the BP network algorithm, which is currently widely used in computer prediction and retrieval, to optimize the detection elements of the instructional resource network sharing platform, so as to achieve the purpose of improving the user experience of the instructional resource network sharing platform [13]. Sun put forward the preliminary idea of applying NN in educational resource management. At the same time, combined with the structural characteristics of NN, an educational resource management system model was designed, a new model of educational resource management was constructed, and its advantages in educational resource management were discussed [14]. Yz et al. took advantage of the multilayer perceptron for nonlinear data processing, and converted the prediction method of vector multiplication of learner characteristics and instructional resource characteristics into the method of inputting the multilayer perceptron, and improved the DN-CBR recommendation model [15]. Bamford et al. used advanced integration theory and integration thought, as well as open-source DSpace and advanced modern technology to integrate, cluster, optimize, and reorganize network instructional resources into a new organic whole, forming a better and more efficient higher new network instructional resources integration system [16]. Based on JavaEE technology and Ajax front-end development technology, Sreethar et al. have implemented a music instructional resource management system in institution of higher learning. Based on the requirements document, a series of functional test cases are designed; in terms of system performance, two stress test schemes for read and write performance are designed [17].

The related literature studies are thoroughly examined in this article, and DCNN technology is discussed. Based on the foregoing, a DCNN-based music instructional resource management platform is proposed and designed. The algorithm in this article takes advantage of the advantages of multilayer perceptron in nonlinear data processing and converts the vector multiplication prediction mode of learner characteristics and instructional resource characteristics into the mode of input multilayer perceptron, thus improving the traditional NN model. Simultaneously, the demand for music instructional resource management in institutions of higher learning is analyzed in depth and detail using the demand analysis tool, and a demand document is created. This article examines the various types of music instructional resources and summarizes resource classification methods that correspond to actual instructional activities. Design each requirement item in detail, and produce design documents based on the requirement documents. The experiments have shown that this system can meet the needs of users while also providing the most educational benefits.

## 3. Methodology

### 3.1. Resetting and Integrating Music Instructional Resources

DL network is extended from NN. NN is a mathematical model that tries to imitate the design of the human brain system, and it has better information storage and processing ability. It is a complex calculation method to simulate neurons and neuronal connection structure of the human brain [18]. NN technology mainly takes the workflow of the human nerve as the design model and calculates by using the way of human nerve processing related content. Deep belief network is a kind of NN, which is initialized layer by layer by an unsupervised learning algorithm. The time complexity of optimizing the weight of the deep belief network and the linear relationship between the network scale and depth, starting from the simple single-layer problem, solve the problem of a complex deep layer constructed by a single layer, and reduce the training difficulty of the DL network. As a new research field of machine learning, the purpose of DL is to study how to automatically extract multilayer features from data. In DL, CNN is one of the classic and widely used models. The basic unit of NN is called neuron, and interconnected neurons form a NN. Although only some simple basic operations are performed on each node, they can realize many complicated calculations when connected to different network structures [19]. The connection weight between neurons reflects the connection strength between units, and the representation and processing of information is reflected in the connection relationship of network processing units. It can be used for intelligent control, speech recognition, and other more intelligent content. The essence of NN is to obtain a parallel and distributed information processing function through network transformation and dynamic behaviour, and to imitate the information processing function of the human brain nervous system in different degrees and levels. Because of this important feature, NN adopts a completely different mechanism from traditional artificial intelligence technology, and overcomes the defects of traditional artificial intelligence based on logical symbols in dealing with intuitive and unstructured information. When a pair of networks learn patterns, the activation value of neurons goes from the input layer to the output layer through the middle layer, and the output of neurons in the output layer corresponds to the response of each input pattern network. It has the characteristics of self-adaptation, self-organization, and real-time learning. It can better deal with the problems that the current artificial intelligence cannot solve through the connection between neurons. Choosing a reasonable network model structure plays a very important role in reducing the training times of the network and improving the learning accuracy of the network. Generally speaking, the input layer depends on the specific problem.  Figure 1 shows the DL network model.

Instructional resources are always the foundation of education and the support of quality education. Constantly expanding the instructional resources of music courses and perfecting textbooks are the important guarantee to realize the reform goal of music teaching in the institution of higher learning, and also help to improve the overall quality of college students. Internet technology has the characteristics of sharing and immediacy, so the information resources of online music education have these two characteristics. On the one hand, online music education resources can allow learners with different numbers to browse and learn at the same time, so it has the characteristics of sharing. On the other hand, after the online music education resources are uploaded to the Internet, related customers can inquire about music education resources at anytime and anywhere, which breaks the time and space constraints. In the broad sense of curriculum resources, music curriculum resources not only refer to music teaching materials or music instructional videos, but human factors, especially student factors, are the most important resources. It is the main body of college music teaching and the key to improve the utilization efficiency of curriculum resources. The ultimate goal of college music teaching is to improve college students' music literacy. The ontology of instructional resources represents the knowledge about instructional resources. The ontology mainly includes the types and formats of instructional resources. Among them, the types of instructional resources include handouts, exams, and homework. The format of instructional resources includes text, images, audio, or video. If we want to make better use of online music education resources, we need to constantly develop and utilize them. Therefore, we need to develop and integrate the online music education resources database from three aspects: perfecting the retrieval mechanism of music resources, building self-expanding online music education resources database, and strengthening the standardized management of local resources. The emergence of new media forms rectified the traditional face-to-face communication mode, and the concept of new media was born. In the new era, the media has been applied in the development of all sectors of society, and the education field has also taken the initiative to practice the new media reform route. With the help of the new media platform, it can quickly collect, summarize, sort out, and integrate all kinds of resources. The diversity of educational resources puts forward higher requirements for educators, requiring educators, especially front-line teachers, to screen the most valuable resources in a short time and guide students to make use of network resources correctly and scientifically.

At present, the expansion of educational resources is extremely fast, and it is more and more difficult to classify the massive educational resources. The original artificial classification cannot keep up with the frequency of information transmission, which makes it difficult to find the information users urgently need in a short time, wastes users' time, and also brings obstacles to the further popularization and use of educational resources. Therefore, it is very necessary to integrate the numerous and complicated information resources. The diversity of online music education information resources is mainly manifested in the diversity of its forms, and there are various forms of music education information resources on the Internet. The online music education resources such as pictures, articles, videos, and audio can be expressed in any kind of media supported by digital technology. Therefore, the online music education information resources have the characteristics of diversity in expression forms. The resources that meet the psychological and aesthetic needs of college students are called the best educational resources. During the follow-up teaching of music courses in institution of higher learning, teachers not only impart basic knowledge, but also stimulate students' interest in learning subject knowledge. Under the domination of learning interest, students can gradually form a unique aesthetic view of music. Resources that meet the interests and aesthetic standards of college students are undoubtedly the best educational resources, which can not only impart basic music knowledge, but also enhance college students' interest in music learning. It is the general trend to integrate the network instructional resources and realize the cross-database retrieval of heterogeneous resources. University libraries can become the incomparable builders of this resource pool. This is not only because of the hardware facilities, librarians' quality, academic atmosphere, and readers' needs of university libraries, but also because it can take relevant measures to collect, manage, and integrate university resources. What's more, the nature of the library's work determines that they have the ability to implement the development and integration of the school's resources. In addition, teachers are required to develop and utilize online music curriculum resources from two aspects: the development of music instructional content and the development of a supporting environment for online music teaching. Relevant personnel should pay attention to the establishment of syllabus, instructional design, prototype realization of online music courses and other links, and develop and improve the online instructional environment provided by the construction of software and hardware systems related to online music courses. During the construction of campus culture, we should vigorously publicize the significance of inheriting regional music culture, so as to help college students establish and strengthen their awareness of learning and internalizing regional music culture. At the same time, during the teaching of regional music culture, practice links should be added to strengthen college students' understanding of this kind of educational resources.

### 3.2. Construction of Music Instructional Resource Platform Based on DCNN

The network resources are in a chaotic and disorderly distribution state. The network is a cooperative system for storing, processing, and utilizing these resources. The communication between systems and the full utilization of network resources requires the overall cooperation of all aspects. Therefore, the prerequisite of networking is to adopt a series of standards in resource organization and processing, and realize the standardization of data format, description language, and indexing language. The management platform of music instructional resources is mainly to reset and integrate the instructional resources generated in the process of music teaching, providing convenience for teachers' teaching and students' autonomous learning. The resource integration method based on DCNN mainly consists of two parts. The first part is the technical part, that is, the Arduino device identification program based on CNN, which realizes the classification and identification of Arduino devices through the program. The second part is the part of instructional resources. By collecting and screening the existing instructional resources and making them into videos, the construction of Arduino device instructional resource database is completed. Educational resource management system needs to continuously absorb new educational resources. Provide users with reliable information output. However, when something goes wrong, the educational resource management system is easy to stop working, which brings great losses to users. Therefore, the fault tolerance of the system is more important. In the system deployment architecture, two service sets are clusters, namely, web server cluster and database server cluster. The web server cluster performs session sharing and request distribution through the global load balancer. The database is divided into two parts: the master server and the slave server. The main database server has one instance, which is responsible for all write requests. The integration model of music instructional resources based on DCNN is shown in Figure 2.

The term “resource collection” refers to the process of gathering-related resources from the vast Internet information group and organizing them for users to browse and query based on the needs of music disciplines or fields. Manual collection, automatic collection, and semi-automatic collection are the three methods for gathering resources. The image format must be converted after the image collection and data set construction are completed. This procedure necessitates the conversion of a JPEG image file into a CNN-compatible file format. Educational resources are distributed, stored, and processed in parallel in NN; that is, NN stores educational resources based on the strength of connections between neurons, and educational resource processing is done collectively by network neurons. By downsampling after the convolution layer, the pool layer is primarily used to reduce the dimension of the feature graph and network parameters. Mean pooling and maximum pooling are two common pooling operations. Small changes in the feature map can be ignored by the pool operation, which improves accuracy and effectively avoids overfitting. The activation function for the convolution layer is ReLU. A pool layer is applied after each convolution layer, and the convolution layer is pooled and normalized locally. The output layer's final layer is the full connection layer, which uses the Softmax regression model. The model is trained using this network, and the next section will make appropriate adjustments to the network model based on the experimental results. There are many different types of information resources that various parties collect. The indexed resources are classified according to a certain level to form a systematic classification system, which is based on adhering to standardization. When describing network information resources, we should choose the appropriate metadata format and special software to describe and extract metadata according to our own needs. Storage reliability of instructional resources: data should be processed redundantly, for example, using expensive hardware RAID or distributed mirroring. During the learning process, learners use the Arduino device identification program based on CNN. The identification program tells learners the names of the identified devices and pushes the instructional resources related to the identified devices, including text resources and video resources.

The text matrix *D* ∈ *R*^*n*×*m*^ of instructional resources can be expressed as

(1) $$\begin{array}{c} \left[\begin{array}{cccc} w_{11} & \ldots & w_{1i}\ldots & w_{1m}\\ w_{21} & \ldots & w_{2i}\ldots & w_{2m}\\ \ldots & \ldots & \ldots & \ldots \\ w_{n1} & \ldots & w_{ni}\ldots & w_{nm} \end{array}\right]. \end{array}$$

Here, *m* represents the dimension of the embedding; *n* represents the number of words; and *w*_[*i*, 1 : *m*]_ represents the vector form of the *i* th word. The calculation formula of the feature map is

(2) $$\begin{array}{c} m_{i}=f\left(D^{*}F_{i}+b_{i}\right). \end{array}$$

Here, ^*∗*^ represents the convolution calculation; *b*_*i*_ represents the bias term; and *f*(·) is a nonlinear activation function. Nonlinear factors can be introduced into the model to solve the eigenvectors that are difficult to represent by linear models, and the ReLU function is used in this model. Cross-entropy is a widely used loss function, and this article also uses cross-entropy as a loss function. The formula for cross-entropy is

(3) $$\begin{array}{c} H\left(p,q\right)=-\sum_{x}p\left(x\right)\log\;q\left(x\right). \end{array}$$

When it is used as the loss function of NN, *p* represents the correct answer and *q* represents the predicted value. The smaller the value of cross-entropy, the closer the two probability distributions are, which means the better the constructed NN model. Suppose the feature map obtained in the *t* th convolutional layer is given by

(4) $$\begin{array}{c} M_{t}=\left\{m_{1},m_{2},m_{3},\ldots ,m_{s}\right\}. \end{array}$$

Maximum pooling is used to extract the maximum value in *M*_*t*_; *p*_*i*_ represents the pooling result of the *t*_*i*_ th convolutional layer, which is formally expressed as

(5) $$\begin{array}{c} p_{i}=\max\left(M_{t}\right)=\max\left\{m_{1},m_{2},m_{3},\ldots ,m_{s}\right\}. \end{array}$$

Assuming that there are *m* neurons in the fully connected layer, after the ReLU activation function, a fixed-size vector *s* is obtained, which is the text feature vector of the instructional resource. The calculation formula is

(6) s=ReLUwipi+bi.

Here, *p*_*i*_ represents the output of the instructional resource text information on the pooling layer; *w*_*i*_ represents the weight; and *b*_*i*_ represents the corresponding bias. The characteristic *v*_*j*_ of instructional resource *j* can be expressed as

(7) $$\begin{array}{c} v_{j}=s_{j}+t_{j}. \end{array}$$

Given *M* retrieval targets, the sample input size *X* is

(8) $$\begin{array}{c} {\left\{x^{a}\right\}}_{a=1}^{m}. \end{array}$$

When *x* ∈ *R* and {*c*^*k*^}_*k*=1_^*p*^ ⊂ *R*^1^ is output, it is assumed that the retrieval target parameters in a period of time are discrete *f*(*x*), if this function has

(9) $$\begin{array}{c} f\left(x\right):R^{1}⟶R^{a}. \end{array}$$

Then, the retrieval weight vector *Z*=(*z*_1_, *z*_2_, *z*_3_,…, *z*_*m*_) ∈ *R*^*m*^ and the threshold *θ* accepted by the nodes on a level can satisfy the following formula:

(10) $$\begin{array}{c} c_{k}=f\left(z*x^{k}-\theta \right)=f\left(\sum_{a=1}^{m}Zax_{m}^{k}-\theta \right),\;k=1,2,3,\ldots ,p. \end{array}$$

Select an appropriate resource management and publishing platform. By providing various unstructured databases and traditional relational databases, the platform can facilitate online publishing. At the same time, it can improve the retrieval efficiency and full-text retrieval ability of online publishing of databases to meet the needs of Internet applications. If the system is faced with the problem of network overload, because the storage is distributed, the information resources can be easily allocated. In addition, even if there is a sudden power failure, because the related resources have been stored, the loss is minimal. The robustness of the system is greatly enhanced. At the same time, if the system suddenly fails, because there are two input channels, it can be easily handled by another server. The same is true when processing. Therefore, the fault tolerance of the system is also improved. In the process of DCNN model training in this article, the pictures are converted into TFRecord files, which are used as the initial data input of the network. After processing the image data, DCNN realizes the output of the network model through multilayer convolution and pooling operations. By comparing the error information between the actual output and the expected output, the test accuracy value and error loss function that describe the model are observed and analyzed. With the continuous increase of instructional resources, it may be necessary to add more storage devices to expand the existing storage system, so it is necessary for data storage to have strong scalability. The integrated digital resource system provides users with a single access portal-integrated system, which is used to submit and share resources. The tool used by the user is a simple browser. For the resource integration system, this is a thin client application mode, and the system maintenance only needs the administrator on the background server, without maintaining the front-end application.

## 4. Result Analysis and Discussion

Resetting and integrating resources under the network environment is a systematic work, which needs to orderly represent the external features and content features of resources according to certain steps and procedures, so as to achieve the purpose of ordering resources, facilitate users to use information and effectively transmit information, and realize the coconstruction and sharing of resources. In order to ensure the safe and stable operation of the system, experiments are carried out in this chapter to test the feasibility of the proposed method. As the collected data has both structured data and unstructured data, it is necessary to preprocess the data. Preprocessing should classify the data, and different processing methods should be selected for different classifications. The test environment of this chapter is shown in Table 1.

The training phase of the model is a process of constantly changing parameters and optimizing. This process continues until the output data value converges and tends to a stable state, or the iteration number ends, and the model training ends. At this time, a classification model can be obtained and used in the image classification process. The model training situation is shown in Figure 3.

In this article, MAE (mean absolute error) and accuracy rate are selected for testing, and then, the results are compared with fuzzy clustering algorithm [20] and BP algorithm. The MAE of different algorithms is shown in Figure 4. The accuracy of different algorithms is shown in Figure 5.

It can be seen that the accuracy of this algorithm is high and the MAE is low. By taking a unified management platform as the core, this article resets, optimizes, and integrates all kinds of music education resources, which improves the problems that the previous educational resources management was designed from the perspective of single function: the functions cannot be combined with each other, resulting in resource management difficulties and incompatible resources. It maximizes the value of educational resources. Test the operation of the system. The operation of different systems is shown in Figure 6.

It can be seen from the data trend in Figure 6 that the system in this article takes relatively little time and runs well. The test results show that the system basically achieves the expected purpose. In this article, recall, precision, and similarity are selected as three indicators, and five experiments are conducted, respectively. The data results of the indicators in this article are shown in Table 2.

Experiments show that the accuracy of the proposed algorithm is improved by about 6% compared with the fuzzy clustering algorithm. At the same time, the stability of this system can reach 96.14%. The security of the application layer of the system is considered from three aspects: ① enhancing the security of the application server system. ② Adopt identity authentication mechanism to ensure the reliability of application. ③ Adopt data encryption technology and anti-virus software to ensure the security of application. Because the system faces a wide range of people, it needs to have certain stability. The stability of the system is tested below, and the test results are shown in Figure 7.

From the stability test results of the system, it can be seen that the system in this article can still maintain a certain stability in the case of a large amount of operation. This shows that the music instructional resource platform constructed in this article has certain reliability and practicability. In order to verify the reliability of the method proposed in this article, several experiments are carried out in this chapter. The experiments show that the accuracy of the proposed algorithm is improved by about 6% compared with the fuzzy clustering algorithm. At the same time, the stability of this system can reach 96.14%. The results show that the music instructional resource platform constructed in this article has certain reliability and practicability.

## 5. Conclusions

A music resource management system is proposed in the context of educational information technology development. The foundation of information teaching is educational resources. This article creates a model of music instructional resource management system, constructs a new model of educational resource management, and discusses its benefits in educational resource management based on the structural characteristics of DCNN. The overall goal, design principle, overall structure, and interface design of the system are all discussed in this article. The algorithm in this article takes advantage of the advantages of multilayer perceptron in nonlinear data processing and converts the vector multiplication prediction mode of learner characteristics and instructional resource characteristics into the mode of input multilayer perceptron, thus improving the traditional NN model. The experiments show that when compared to the fuzzy clustering algorithm, the proposed algorithm improves accuracy by about 6%. At the same time, this system's stability can reach 96.14 percent. The music instructional resource platform developed in this article has a high level of dependability and usability. The music resource integration system has a number of features that can be used to meet the needs of a variety of applications, including submission, preservation, management, and publication of educational resources. It has the potential to provide a workable plan for the management of instructional resources in a variety of disciplines. Although this article makes a relatively comprehensive research on the management platform of music instructional resources through various technologies, there are still some shortcomings. Many follow-up work, such as the function expansion and resource integration of the network instructional resource integration system, need to be further studied and discussed.

## Figures and Tables

**Figure 1:** DL network model.

**Figure 2:** The integration model of music instructional resources based on DCNN.

**Figure 3:** Model training.

**Figure 4:** Comparison of accuracy results of different algorithms.

**Figure 5:** MAE comparison of algorithms.

**Figure 6:** Comparison of operation conditions of different systems.

**Figure 7:** Stability of the system.

**Table 1:** Test environment.

Environment	Category	Set up
Hardware environment	CPU	Dikaryon
	RAM	512 MB
	Hard disc	1 TB
	Network card	100/1000 self-adaption

Software environment	System	Windows
	Browser	IE6.0 up

**Table 2:** Experimental results of each index.

Number of experiments	Recall ratio	Precision ratio	Similarity
1	89.64	88.61	0.164
2	88.79	90.31	0.157
3	90.12	90.02	0.172
4	89.95	89.97	0.153
5	91.34	90.18	0.159

## Data Availability

The data used to support the findings of this study are available from the corresponding author upon request.
